# LncRNA ANRIL affects the sensitivity of ovarian cancer to cisplatin via regulation of let-7a/HMGA2 axis

This article has been retracted.

**DOI:** 10.1042/BSR20182101

**Published:** 2019-07-05

**Authors:** Jin-Tian Miao, Jian-Hua Gao, Yong-Qian Chen, Hong Chen, Hao-Yi Meng, Ge Lou

**Affiliations:** 1 Department of Gynecology, The Affiliated Tumor Hospital of Harbin Medical University, Harbin, Heilongjiang, China; 2 Department of Gynecology, The First Affiliated Hospital of Harbin Medical University, Heilongjiang, China

**Keywords:** ANRIL, cisplatin, HMGA2, let-7a, ovarian cancer, sensitivity

## Abstract

This paper tried to explore ANRIL expression in ovarian cancer and how it affects cisplatin-sensitivity of ovarian cancer cells via regulation of let-7a/high-mobility group protein A2 (HMGA2) axis. qRT-PCR was used to detect ANRIL and let-7a levels in ovarian cancer tissues and cell lines (SKOV3 and SKOV3/DDP). Then cells were randomly assigned into Blank, negative control siRNA, ANRIL siRNA, let-7a inhibitor, and ANRIL siRNA+let-7a-inhibitor groups. CCK-8 assay was applied for assessing cell viability of cells treated with different concentrations of cisplatin. Flow cytometry was employed to test cell apoptosis rate. qRT-PCR and Western blot were performed for related molecules detection. Nude mice transplanted with SKOV3/DDP cells were used to confirm the effects of ANRIL siRNA on the cisplatin-sensitivity. Ovarian cancer tissues and cisplatin-resistant cells had increased ANRIL expression and decreased let-7a expression, and those patients with higher clinical stage and pathological grade showed higher ANRIL and lower let-7a. Dual-luciferase reporter-gene assay confirmed the targeting relationship between ANRIL and let-7a, and between let-7a and HMGA2. The cell viability and cisplatin IC_50_ were decreased in ANRIL siRNA group exposed to different concentrations of cisplatin, with enhanced apoptosis, as well as elevated let-7a and declined HMGA2, which would be reversed by let-7a inhibitor. Meanwhile, ANRIL down-regulation enhanced the inhibitory effect of cisplatin on tumor growth of nude mice and reduced tumor weight. Silencing ANRIL expression reduced HMGA2 expression to promote the apoptosis and improve cisplatin-sensitivity of ovarian cancer cells via up-regulating let-7a expression.

## Introduction

Ovarian cancer, a very prevalent gynecologic malignancy, is characterized by early-onset metastasis, poor prognosis and multidrug resistance (MDR), with epithelial ovarian cancer being the most common type globally [1,2]. According to statistics, the average 5-year survival rate of ovarian cancer patients is ∼45.6% [3], and ovarian cancer becomes the fifth major cause of female death worldwide [4]. At present, the primary therapy for ovarian cancer is still surgery combined with chemotherapy, with cisplatin being one of the most common chemotherapeutic drugs [5]. However, MDR during chemotherapy is the main tackle of treatment failure, severely affecting the life quality of patients [6]. Therefore, it is imperative to understand the mechanism of drug resistance in ovarian cancer and thereby improve the prognosis of ovarian cancer patients.

Long non-coding RNA (lncRNA) consists of over 200 nucleotides and is mainly distributed in nucleus or cytoplasm, and it can affect a variety of biological processes by regulating the expression of genes [7]. LncRNA ANRIL (antisense non-coding RNA in the INK4 locus) is on the 9q21.3 region of chromosome, which was initially found and named by Pasmant et al*.* in a genetic study of melanoma deletion strains [8]. ANRIL has been found excessively expressed in several different malignant tumors, such as liver cancer [9], lung cancer [10], and esophageal cancer [11], acting as an oncogene. As revealed by Qiu et al. [12], elevated ANRIL constitutes an indicator of the poor prognosis of ovarian cancer patients, whereas ANRIL inhibition could block the invasion and migration of ovarian cancer cells. However, there are limited data concerning the effect of ANRIL on the sensitivity to cisplatin in ovarian cancer. Recently, it has been demonstrated that ANRIL has a bearing on the chemosensitivity of tumors. For example, a study reported that silencing ANRIL could hinder the development of MDR in gastric cancer cells [13], which could also up-regulate microRNA let-7a to inhibit tumorigenicity and enhance the chemosensitivity of nasopharyngeal carcinoma cells to cisplatin [14]. It is particularly worth mentioning here that there is a targeting relationship between ANRIL and let-7a, and between let-7a and HMGA2, as confirmed by the analysis of our dual-luciferase reporter-gene assay. To our knowledge, let-7, as the second-discovered miRNA family, can participate in a variety of biological processes, such as the growth, differentiation, and proliferation of cells [15,16]. Also, there was evidence demonstrating that the obviously declined let-7a expression was found in ovarian cancer [17]. In addition, the high-mobility group protein A2 (HMGA2) is a member of the high-mobility group protein family, playing an important role in carcinogenesis and the chemotherapeutic drug resistance of cells [18]. In the study of Xiao et al. [19], let-7a was discovered able to specifically regulate HMGA2 to influence pancreatic cancer cells’ sensitivity to chemotherapeutic drugs. And, it could also modulate the expression of HMGA2 in ovarian cancer cells through targeted regulation [20]. Along these clues, we hypothesized that ANRIL may regulate the let-7a/HMGA2 axis to some extent to influence the cisplatin-sensitivity of ovarian cancer cells.

Therefore, through *in vivo* and *in vitro* experiments, we aimed to investigate whether ANRIL could affect the cisplatin-sensitivity of ovarian cancer by regulating let-7a/HMGA2 axis, so as to look for a novel strategy to alleviate the cisplatin resistance in ovarian cancer.

## Materials and methods

### Study subjects

From January 2016 to December 2017, a total of 86 epithelial ovarian cancer patients (with the mean age of 50.23 ± 11.57 years) were admitted to our hospital and undertaken surgical treatment. All those patients never received chemotherapy or radiotherapy prior to operation, and among them, 50 cases were serous cystadenocarcinoma of the ovary, while 36 cases were other types. According to the pathological grading, 37 patients were in G_1_-G_2_ and 49 cases in G_3_; meanwhile, based on clinical cancer staging [22], there were 35 cases in stage I–II and 51 cases in stage III–IV. In addition, normal ovarian tissues were collected from 35 patients who underwent hysterectomy with resection of bilateral ovaries and fallopian tubes because of hysteromyoma or adenomyosis. All tissue samples were examined pathologically and cryopreserved in liquid nitrogen at −80°C.

### Ovarian cancer cell culture

The normal human ovarian surface epithelial cells (HOSEPiCs) and human ovarian cancer cells (cisplatin-sensitive strain SKOV3 and cisplatin-resistant strain SKOV3/DDP) were provided by the Cell Bank of Chinese Academy of Sciences in Shanghai and cultured in RPMI1640 containing 10% fetal bovine serum, in an incubator (37°C, 5% CO_2_) (Thermo Forma, U.S.A.). Cells were passaged when they reached ∼90% confluency.

### Transfection experiments

At the logarithmic growth phase, SKOV3 and SKOV3/DDP cells were collected and randomly divided into five groups, Blank group (cells without transfection), negative control (NC) siRNA group (cells transfected with ANRIL NC siRNA), ANRIL siRNA group (cells transfected with ANRIL siRNA), let-7a mimic group (cells transfected with let-7a mimic), and ANRIL siRNA+ let-7a-inhibitor group (cells co-transfected with ANRIL siRNA and let-7a inhibitor). ANRIL siRNA and let-7a inhibitor/mimic were bought from Shanghai GenePharma Co., Ltd. When cell confluence reached 70%, transfection was performed according to the manufacturer’s instructions on the Lipofectamine 2000 kit (Invitrogen). All sequences used are provided in Supplementary Table S1.

### Cisplatin-sensitivity detected by CCK-8 assay

Different groups of SKOV3 and SKOV3/DDP cells were inoculated onto 96-well plate respectively by 100 μl/well with five replicates. Next, cisplatin of different concentrations (0, 1.25, 2.5, 5, 10, 20, 40, and 80 μM) [23] (SelleckBio, U.S.A.) were added into each well for continued culture for 72 h, followed by the addition of CCK8 solution at 10 μl/well and followed by another 4 h of incubation. Finally, a microplate reader was used to read the OD values at a wavelength of 450 nm, cell survival curve was drawn, and 50% inhibitory concentration (IC_50_) of cisplatin was calculated accordingly.

### Cell apoptosis detected by flow cytometry

After removing the culture medium, SKOV3 and SKOV3/DDP cells were washed with PBS buffer for two times, digested by 0.25% trypsin, harvested into centrifuge tube, and centrifuged at the rate of 1000 rpm for 3 min. Next, Annexin V Binding Solution was used to make single cell suspension with the cell density of 10^6^ cells/ml. Later, 100 μl single cell suspension was taken and incubated with 5 μl of Annexin V-FITC and 5 μl of PI solution was added for 15 min at room temperature without exposure to light. Eventually, 400 μl Annexin V binding solution was used for dilution and a flow cytometer (BD FACSCalibur) to detect cell apoptosis rate.

### Dual-luciferase reporter-gene assay

ANRIL was inserted into wild-type ANRIL-3′UTR-WT plasmid and mutant-type ANRIL-3′UTR-MUT plasmid to make ANRIL dual-luciferase reporter gene plasmids. Meanwhile, wild-type HMGA2-3′UTR-WT plasmid and mutant-type HMGA2-3′UTR-MUT plasmid were also constructed. SKOV3 cells collected at the logarithmic growth phase were inoculated onto 96-well plate, and transfection was performed with Lipofectamine 2000 kit when cell confluence reached ∼70%. Before transfection, ANRIL-3′UTR-WT or HMGA2-3′UTR-WT plasmid was mixed with let-7a mimic/NC plasmid. At the same time, the control wells (ANRIL-3′UTR-WT+NC/HMGA2-3′UTR-WT+NC and ANRIL-3′UT R-MUT+ let-7a mimic/HMGA2-3′UTR-MUT+ let-7a mimic) were also needed. At last, luciferase activity was tested by Dual-Glo® Luciferase Assay System (Promega, U.S.A.). *Renilla* luciferase activity was normalized to the corresponding firefly luciferase activity. All sequences used are provided in Supplementary Table S1.

### qRT-PCR

Cells were collected to extract total RNA with the RNA extraction kit (Omega, U.S.A.). Then, RNA purity and concentration were determined with an ultraviolet spectrophotometer (UV-1800, Japan) and RNA integrity was observed after the agarose gel electrophoresis. Primers were designed by using the Primer 5.0 software and all primers were synthesized by Sangon Biotech (Shanghai) Co. Ltd (Supplementary Table S1). The reverse-transcription of total RNA into cDNA was achieved by a PrimescriptTM RT reagent kit (Takara, Japan). The SYBR® premix Ex Taq TM PCR kit (Takara Biotechnology (Dalian) Co., Ltd.) was used for qRT-PCR and the relative expression of genes was calculated by using the 2^−ΔΔ*C*^t method with U6 and GAPDH as the internal controls.

### Western blot analysis

Cells were placed into lysate for the extraction of total proteins, which were centrifuged at the rate of 12000 rpm for 15 min before collecting the supernatant for SDS-PAGE electrophoresis. The proteins separated by electrophoresis were transferred to the nitrocellulose filter by electric transfer, and the filter was blocked for 1 h in 5% skimmed milk-PBS solution. Next, primary antibody HMGA2 (ab32109, 1:1000 dilution, Abcam), Caspase-3 (ab2302, 1:1000 dilution, Abcam), Bcl-2 (ab182858, 1:1000 dilution, Abcam), and Bax (ab53154, 1:1000 dilution, Abcam) was added for overnight reaction at 4°C. The filter was washed thrice with PBS buffer before 1 h of incubation at room temperature with horseradish peroxidase conjugated secondary antibody. Subsequently, the filter was rinsed again for three times with PBS buffer before development by the enhanced chemiluminescence (ECL) method. The gray value ratio of target bands to the reference band was used to evaluate the relative expression level of proteins, with GAPDH as the internal reference.

### Nude mice transplanted with human ovarian cancer cells

BALB/c-nu nude mice of 4-week-age were subcutaneously injected with SKOV3/DDP cells those transfected with ANRIL siRNA/NC siRNA. When the average tumor diameter was at least 0.5 cm, ANRIL siRNA and NC siRNA xenografts were randomly divided into cisplatin-treated group and normal saline (NS)-treated group (*n*=8 in each group). To be specific, mice in the cisplatin-treated group were treated intraperitoneally with cisplatin (5 mg/kg) every 4 days for 28 days, while those in the NS-treated group were given 0.2 ml NS. The tumor volume was calculated according to the following formula (L × W^2^)/2 after measuring the length (L) and width (W) with calipers. After the experiment, the mice were killed and their tumors were taken out for mass weighing. The excised tumors were fixed at 4°C in paraformaldehyde and embedded in paraffin. Tumors sections were used for HE staining and immunohistochemistry analyses.

### Statistical analysis

All experiments were repeated for three times. The software SPSS 21.0 was used for data analysis. Measurement data were expressed as mean ± standard deviation ($\bar{\text{x}}\pm \text{s}$). The comparison was performed with Student’s *t* test, One-Way ANOVA, or conducted by using Tukey’s post-hoc test. *P*<0.05 suggested the statistically significant.

## Results

### Expression of ANRIL and let-7a in ovarian cancer tissues and cisplatin-resistant cell lines

As for ovarian tissues shown in Figure 1, the ovarian cancer tissues had apparently higher ANRIL expression and lower let-7a expression than its adjacent normal tissues (all *P*<0.05). Additionally, compared with normal HOSEPiCs, the cisplatin-sensitive and cisplatin-resistant cell lines (SKOV3 and SKOV3/DDP cells) had significantly increased ANRIL expression and decreased in let-7a expression (all *P*<0.05). Moreover, the SKOV3/DDP cells were higher in ANRIL but lower in let-7a than the SKOV3 cells (all *P*<0.05). According to the analysis of clinicopathological features demonstrated in Table 1, ANRIL and let-7a expression levels had no correlations to the age, pathological type, and tumor size (all *P*>0.05), but were closely associated with clinical staging and pathological grading of patients (all *P*<0.05). Especially, ovarian cancer patients with higher clinical stage and pathological grade had higher expression of ANRIL and lower expression of let-7a (all *P*<0.05).

**Figure 1:** Expressions levels of ANRIL and let-7a in ovarian cancer tissues and cisplatin-resistant cell lines The expression levels of ANRIL(**A**) and let-7a (**B**) in ovarian cancer and adjacent tissues. The expression levels of ANRIL (**C**) and let-7a (**D**) in HOSEPiCs, SKOV3, and SKOV3/DDP cell lines; *, *P*<0.05 compared with normal HOSEPiCs; #, *P*<0.05 compared with SKOV3 cells.

**Table 1:** The correlation of LncRNA-ANRIL and let-7a expressions to the clinicopathological features of ovarian cancer patients

Clinicopathological features	*n*	ANRIL	*P*	let-7a	*P*
Age			0.612		0.564
≥50	48	3.54 ± 0.43		0.42 ± 0.07	
<50	38	3.49 ± 0.48		0.41 ± 0.09	
Pathological type			0.841		0.549
Ovarian serous cystadenocarcinoma	50	3.51 ± 0.47		0.42 ± 0.08	
Other	36	3.53 ± 0.43		0.43 ± 0.07	
Tumor size			0.837		0.250
≥10	41	3.53 ± 0.47		0.41 ± 0.08	
<10	45	3.51 ± 0.43		0.43 ± 0.08	
Clinical staging			<0.001		<0.001
I–II	35	3.10 ± 0.31		0.49 ± 0.07	
III–IV	51	3.81 ± 0.27		0.37 ± 0.04	
Pathological grading			<0.001		<0.001
G_1_–G_2_	39	3.14 ± 0.32		0.48 ± 0.07	
G_3_	47	3.83 ± 0.27		0.36 ± 0.04	

### Effect of ANRIL on the sensitivity of SKOV3 and SKOV3/DDP cells to cisplatin

In terms of SKOV3 cells displayed in Figure 2A,B, the cell viability and cisplatin IC_50_ were decreased in ANRIL siRNA and let-7a mimic groups compared with the Blank group after treated with different concentrations of cisplatin (all *P*<0.05). In the meantime, ANRIL siRNA+ let-7a-inhibitor group had dramatically increased cell viability and cisplatin IC_50_, as compared with the ANRIL siRNA group (all *P*<0.05). Additionally, we also explored whether ANRIL can restore the DDP sensitivity in DDP-resistant cells (SKOV3/DDP cells). As illustrated in Figure 2C,D, ANRIL siRNA and let-7a mimic could reduce the viability of SKOV3/DDP cells and IC_50_ of cisplatin (all *P*<0.05), while let-7a inhibitor was able to reverse the effect of ANRIL siRNA on improving cisplatin-sensitivity. Given the above, we may conclude that inhibiting ANRIL could improve the cisplatin sensitivity of ovarian cancer cells and let-7a inhibitor had the opposite effect.

**Figure 2:** Effect of ANRIL on the cisplatin sensitivity The effect of ANRIL on the cisplatin sensitivity of SKOV3 (**A,B**) and SKOV3/DDP (**C,D**) cells observed after CCK-8 assay. *, *P*<0.05 compared with the Blank group; #, *P*<0.05 compared with the ANRIL siRNA group; &, *P*<0.05 compared with the let-7a-inhibitor group.

### Effect of ANRIL on the apoptosis of SKOV3 and SKOV3/DDP cells

In SKOV3 and SKOV3/DDP cells (Figure 3), the NC siRNA group had no significant difference from the Blank group in the cell apoptosis rate (*P*>0.05); however, the ANRIL siRNA and let-7a mimic groups had apparently increased apoptosis rate (all *P*<0.05). In addition, the cell apoptosis rate in the ANRIL siRNA + let-7a-inhibitor group was remarkably lower than the ANRIL siRNA group (*P*<0.05). Besides, we detected the protein levels of classic apoptotic markers in SKOV3 and SKOV3/DDP cells. As expected, western blot analysis showed that ANRIL siRNA and let-7a mimic markedly decreased the expression levels of Caspase-3, while the ratio of Bcl-2/Bax was increased (all *P*<0.05). The expression levels of Caspase-3 in the ANRIL siRNA+ let-7a-inhibitor group was remarkably increased and the ratio of Bcl-2/Bax was decreased as compared with the ANRIL siRNA group (*P*<0.05).

**Figure 3:** The effect of ANRIL on the apoptosis of SKOV3 and SKOV3/DDP cells (**A**–**D**) Cell apoptosis in SKOV3 and SKOV3/DDP cells detected flow cytometry; (**E,F**) Apoptosis-related proteins (Caspase-3, Bax, and Bcl-2) were detected by western blotting in SKOV3 (E,**G**) and SKOV3/DDP (F,**H**) cells; *, *P*<0.05 compared with the Blank group; #, *P*<0.05 compared with the ANRIL siRNA group; &, *P*<0.05 compared with the let-7a-inhibitor group.

### The targeting relationship among let-7, ANRIL, and HMGA2

By using the website http://starbase.sysu.edu.cn/index.php (Figure 4A), we found that ANRIL can specifically regulate let-7a, and the binding site of let-7a to HMGA2 was also predicted with the software Target Scan (Figure 4B). According to the results of dual-luciferase reporter gene assay, let-7a mimic had no obvious effect on the luciferase activity of ANRIL-MUT and HMGA2-MUT (all *P*>0.05), but it can effectively reduce the luciferase activity of ANRIL-WT and HMGA2-WT (*P*<0.05, Figure 4C,D). All those results indicated that there was reciprocal repression between ANRIL and let-7a, and between let-7a and HMGA2.

**Figure 4:** LncRNA-ANRIL and let-7a interact with and suppress the expression of each other (**A,B**) Schematic representation of the predicted target site for let-7a in lncRNA-ANRIL (A), and for HMGA2 in let-7a; (**C,D**) Relative luciferase activities of luciferase reporters bearing wild-type or mutant-type lncRNA-ANRIL/HMGA2 following transfection with the indicated let-7a mimic or mimic NC.

### Effect of ANRIL on let-7a/HMGA2 axis

As shown in Figure 5, ANRIL and HMGA2 were down-regulated and let-7a was up-regulated in SKOV3 and SKOV3/DDP cells in the ANRIL siRNA and let-7a mimic groups (all *P*<0.05), as compared with the Blank group. No alterations were found between Blank group and NC siRNA in these molecules (all *P*>0.05). Moreover, with ANRIL siRNA group as the baseline, ANRIL siRNA+ let-7a-inhibitor group presented obvious increases of ANRIL and HMGA2, and remarkable decrease of let-7a (all *P*<0.05).

**Figure 5:** The expression levels of ANRIL, let-7a, and HMGA2 in SKOV3 and SKOV3/DDP cells (**A,B**) The expression of ANRIL and let-7a in SKOV3 cells detected by qRT-PCR; (**C,D**) the protein expression level of HMGA2 in SKOV3 cells determined by Western-blot; (**E,F**) the expression of ANRIL and let-7a in SKOV3/DDP cells detected by qRT-PCR; (**G,H**) the protein expression level of HMGA2 in SKOV3/DDP cells determined by Western-blot; *, *P*<0.05 compared with the Blank group; #, *P*<0.05 compared with the ANRIL siRNA group; &, *P*<0.05 compared with the let-7a-inhibitor group.

### The growth of transplanted tumor in nude mice

The experiment in nude mice showed that compared with mice in the NC siRNA+NS group, those in the ANRIL siRNA+NS, NC siRNA+cisplatin, and ANRIL siRNA+cisplatin groups were slowed down in tumor growth and reduced in tumor weight and the positive rate of HMGA2 (all *P*<0.05, Figure 6). Among these groups, ANRIL siRNA+cisplatin group showed most obvious inhibitory effect regarding the tumor growth, and nude mice in this group had significantly lower tumor volume and weight and the positive rate of HMGA2 than mice in ANRIL siRNA+NS group and NC siRNA+cisplatin group (all *P*<0.05).

**Figure 6:** ANRIL siRNA increased cisplatin sensitivity in xenograft nude mice (**A**) Representative photographs of tumors in nude mice; (**B**) images are included to identify and define tumor histology; (**C,D**) The tumor growth curve (**C**) and tumor weight (**D**) of transplantation tumor of nude mice; (**E,F**) Expression levels of HMGA in each treatment group. Positive cells are stained brown. Quantified protein levels (area %) in representative xenograft tumors are shown; *, *P*<0.05 compared with the NC siRNA+NS group; #, *P*<0.05 compared with the ANRIL siRNA+NS group; &, *P*<0.05 compared with the NC siRNA+cisplatin group.

## Discussion

Firstly, we found the increased ANRIL and decreased let-7a in both ovarian cancer tissues and cisplatin-resistant cell lines, especially in those patients with high-clinical stage and high-pathological grade. Several lines of previous studies have the similar results as ours, for instance, the up-regulated ANRIL was observed in ovarian cancer patients, which was associated with major clinicopathological features of ovarian tumor, and predicted the poor prognosis [12]. Meanwhile, the down-regulation of let-7a in ovarian cancer tissues had a significant correlation to prognosis [17], suggesting that ANRIL may have an important effect as an oncogene, while let-7a might play an anti-oncogenic role in ovarian cancer. Evidence also revealed the involvement of hypoxia-inducible factor 1α (HIF-1α) in the up-regulation of ANRIL in osteosarcoma under the condition of hypoxia [24]. It is known to all that hypoxia can be found in the majority of solid tumors [25], and HIF-1α takes part in the occurrence, progression, and drug-resistance of tumors by regulating gene transcription and expression [26]. More importantly, HIF-1α has been suggested to be abnormally increased expression in ovarian cancer tissues [27,28], and inhibiting HIF-1α could improve the cisplatin-sensitivity of ovarian cancer cells [29], indicating that ANRIL over-expression in ovarian cancer cells may be closely related to the activation of HIF-1α. Through dual-luciferase reporter gene assay analysis in our research, let-7a was identified as the target gene of ANRIL. Actually, ANRIL has been previously proved to specifically inhibit the expression of let-7a in tumors, including prostate cancer [30] and nasopharyngeal carcinoma [14], showing that let-7a reduced expression in ovarian cancer may be affected by the regulation of ANRIL. In addition, we found ANRIL was higher and let-7a was lower in cisplatin-resistant cells (SKOV3/DDP) as compared with cisplatin-sensitive cells (SKOV3), suggesting that ANRIL may target let-7a to affect the cisplatin resistance of ovarian cancer cells.

Moreover, SKOV3 and SKOV3/DDP cells were selected for transfection *in vitro*. According to the results, silencing ANRIL could reduce the cell viability and cisplatin IC_50_, while inhibiting let-7a would lead to completely opposite tendency. Consistent with our finding, the study by Lan et al. [13] also reported that ANRIL knock-out can reduce cisplatin IC_50_ and increase gastric cancer cells’ chemosensitivity by modulating the expression of MDR-related genes, like *MDR1* and *MRP1*. Liu et al. [31] revealed that LncRNA NEAT1/let-7a-5p axis can target Rsf-1 to regulate Ras-MAPK signaling pathway, and thereby modulating the cisplatin-sensitivity of nasopharyngeal carcinoma. In our experiment, let-7a inhibitor effectively reversed the effect of ANRIL siRNA on improving cisplatin-sensitivity, suggesting that silencing ANRIL may enhance the cisplatin-sensitivity of ovarian cancer cells by regulating the expression in its target gene let-7a. And after knockdown of ANRIL, the apoptosis of SKOV3 and SKOV3/DDP was significantly increased, while inhibition of let-7a resulted in the decreased apoptosis. In agreement, silencing ANRIL can inhibit the proliferation and promote the apoptosis of nasopharyngeal carcinoma cells through up-regulation of its target gene let-7a, eventually improving the chemosensitivity to cisplatin, as reported by Dong J et al. [32]. Silencing ANRIL can suppress cell proliferation, promote cell apoptosis, and reduce the expression of drug transporter MRP1 and ABCC2, thus enhancing the cisplatin-sensitivity of oral squamous cell carcinoma cells [33]. All those findings provided the possibility that ANRIL siRNA can reverse the drug resistance probably by increasing let-7a and decreasing the downstream genes, which can induce apoptosis initiation, enhance the damaging effect of cisplatin on tumor cells, and promote cisplatin-induced cell apoptosis.

Furthermore, to investigate the molecular effect of ANRIL inhibition on the cisplatin-sensitivity of ovarian cancer cells, we also demonstrated that HMGA2 is the target gene of let-7a, and silencing ANRIL led to elevated let-7a but declined HMGA2, but inhibiting let-7a gave rise to the contrary results. In accordance with the pancreatic cancer cells, let-7a was found to specifically down-regulate HMGA2 to improve the chemosensitivity [19]. As reported by Agostini et al. [34], let-7a were inversely correlated with HMGA2 expression in squamous cell carcinoma of the vulva, and at the meantime, Motoyama et al. [35] also found HMGA2 was negatively regulated by the let-7 miRNA family in human gastric cancer. Moreover, Chen et al. [36] reported that let-7a could down-regulate the level of HMGA2, leading to an increased apoptosis in Ton cells. In the study of Dong et al. [32], HMGA2-FOXL2 pathway facilitated the invasion, migration, and epithelial-to-mesenchymal transition of chemo-resistant gastric cancer cells. Also, the highly expressed HMGA2 could increase the drug resistance of pancreatic cancer to chemotherapeutic drugs, as exhibited by Dangi-Garimella et al. [37]. Due to its characteristics, HMGA2 is regarded as an oncogene, and HMGA2 protein AT-hook2 has two phosphorylation sites, serine at which can be phosphorylated by cyclin/CDKs at the beginning of S phase and during G_2_/M phase of the cell cycle, so it can influence cell differentiation and proliferation [38,39]. More importantly, HMGA2 can promote the malignant transformation of ovarian cancer cells, advance cancer cell invasion, and metastasis, and facilitate the growth and proliferation of ovarian cancer cells [40]. Meanwhile, silencing HMGA2 can inhibit the proliferation of ovarian cancer cells and induce cell-cycle arrest at the G_1_ phase and increase cell apoptosis [41]. ANRIL has been identified to be selectively binding with PRC2 complexes to execute histone modifications at specific loci, which indicated that ANRIL may function as the ideal regulator for the epigenetic transcriptional repression [42]. For example, ANRIL could not only interact with SUZ12 (a subunit of the PRC2) and recruit the complex to inhibit the expression of p15 (INK4B), a well-known tumor suppressor gene [8,43,44], but also work in concert with other epigenetic regulators, such as p300 (a histone acetylator), and EZH2 (a histone methyltransferase component of the PRC2 complex) [45,46]. More importantly, previous studies have found that the oncogene HMGA2 may be one of the most important targets up-regulated by the mutations of PRC2 components and encourages the development of HMGA2-targeted therapy for patients with cancers [47,48]. The above evidence suggested that silencing ANRIL could promote ovarian cancer cell apoptosis, increase cisplatin-induced cell apoptosis and improve cisplatin-sensitivity by binding with PRC2 complexes to inhibit HMGA2. Lastly, we further constructed the nude mice models with transplanted tumor to confirm the function of ANRIL *in vivo*. Consequently, ANRIL down-regulation strengthened the inhibitory effect of cisplatin on tumor growth, showing that silencing ANRIL can also enhance cisplatin-induced cytotoxicity and enhance cisplatin sensitivity *in vivo*.

In summary, our study found the up-expression of ANRIL in ovarian cancer tissues and drug-resistant cells, and silencing ANRIL could increase let-7a to further reduce HMGA2, which can promote the apoptosis and improve the cisplatin sensitivity of ovarian cancer cells. Therefore, this strategy provides an alternative therapeutic target for conquering cisplatin-resistance in ovarian cancer.

## Supporting information

**Supplemental Table S1:** Sequences used in the present study

## Abbreviations

HIF-1α: hypoxia-inducible factor 1α
HMGA2: high-mobility group protein A2
HOSEPiCs: human ovarian surface epithelial cells
lncRNA: long non-coding RNA
MDR: multidrug resistance
NC: negative control
NS: normal saline
OD: optical density
qRT-PCR: real-time quantitative reverse transcription polymerase chain reaction
